# Association between serum vitamin D levels and the risk of kidney stone: evidence from a meta-analysis

This article has been retracted.

**DOI:** 10.1186/s12937-016-0148-y

**Published:** 2016-03-31

**Authors:** Hai Wang, Libo Man, Guizhong Li, Guanglin Huang, Ning Liu

**Affiliations:** Department of Urology, Beijing Jishuitan Hospital, No. 31, East Xinjiekou Street, Xicheng District, 100035 Beijing, PR China

**Keywords:** Serum, Vitamin D level, Kidney stone, Meta-analysis

## Abstract

**Background:**

Many epidemiological studies have conducted to evaluate the association between serum vitamin D levels and the risk of kidney stone. The aim of this study was to summarize the evidence from epidemiological studies between them.

**Methods:**

Pertinent studies were identified by a search of PubMed, Embase, the Cochrane Library, China National Knowledge Infrastructure (CNKI) and China Biology Medical literature up to July 2015. Standardized mean difference (SMD) was conducted to combine the results. Random-effect model was used. Publication bias was estimated using Egger’s regression asymmetry test.

**Results:**

Seven articles involving 451 kidney stone cases and 482 controls were included in this meta-analysis. Our pooled results suggested that kidney stone patients had a significantly higher serum vitamin D level compared with controls [summary SMD = 0.65, 95 % CI = 0.51, 0.79, I^2^ = 97.0 %]. The associations were also significant both in Europe [SMD = 0.35, 95 % CI = 0.17, 0.53] and in Asia [SMD = 1.00, 95 % CI = 0.76, 1.25]. No publication bias was found.

**Conclusions:**

Our analysis indicated that serum vitamin D level in kidney stone patients was significantly higher than that in non-kidney stone controls, both in Europe and Asia populations.

**Electronic supplementary material:**

The online version of this article (doi:10.1186/s12937-016-0148-y) contains supplementary material, which is available to authorized users.

## Introduction

Kidney stone disease is common in the general population with an estimated prevalence of about 3–5 % in femalesand 10–15 % in males [1]. The most common type (about >80 %) is the calcium-based kidney stone, and high urine calcium excretion is a strong risk factor for stone formation [2, 3]. Prior studies had shown that a higher concentration of the active vitamin D metabolite, 1,25-dihydroxyvitamin D, is associated with increased urinary calcium excretion [4, 5], which could lead to increase the risk of stone formation.

Despite vitamin D played an important role of in maintaining bone health, as well as a variety of other physiologic functions [6], many clinicians are reluctant to treat vitamin D deficiency or insufficiency in kidney stone formers because of the theoretical risk of increasing urinary calcium excretion. This reluctance likely derives from the fact that vitamin D is often cited as a risk factor for kidney stones [7]. To date, a number of epidemiologic studies have been published exploring the relationship between serum vitamin D level and kidney stone risk. The aim of this meta-analysis was to (1) assess the association of serum vitamin D levels in kidney stone patients compared with the non-kidney stone controls; and (2) assess heterogeneity and publication bias among the studies we analyzed.

## Methods

### Literature search

Two authors independently searched the databases of PubMed, Embase, the Cochrane Library, China National Knowledge Infrastructure (CNKI) and China Biology Medical literature for relevant articles published before July 2015 using the following search terms: ‘cholecalciferol’ OR ‘ergocalciferol’ OR ‘vitamin*’ AND ‘kidney stone’ OR ‘Urolithiasis’ OR ‘nephrolithiasis’ with written in English or Chinese. In addition, we reviewed references of obtained articles. Disagreements between the two authors were resolved by consensus with a third author.

### Study selection

Studies were eligible for analysis if they met the following criteria: (1) the studies were in case–control or cohort design or cross-sectional design or randomized controlled trials; (2) the exposure was serum vitamin D level; (3) the end point was kidney stone; (4) available mean and standard deviation (SD) of serum vitamin D level or data provided from which mean and SD could be calculated; and (5) unrelated case and control groups or exposed and unexposed groups in cohort study and all subjects from the same temporally and geographically defined underlying population. Accordingly, the following exclusion criteria were also used: (1) reviews and (2) repeated or overlapped publications.

### Data extraction

We extracted data from the included articles, with particular regards to: the last name of the first author, publication year, country of region, study design, study population, age for cases and controls, number of cases and controls, the mean ± SD of serum vitamin D levels, and statistical adjustment for the main confounding or mediating factors.

### Statistical analysis

Pooled measure was performed on the standardized mean difference (SMD) with 95 % CI to assess the strength of association between serum vitamin D level and risk of kidney stone. Random-effects model was used to combine study-specific SMD (95 % CI), which considers both within-study and between-study variation [8]. The Q test and I^2^ of Higgins and Thompson [9] were used to assess heterogeneity among included studies. I^2^ describes the proportion of total variation attributable to between-study heterogeneity as opposed to random error or chance, with suggested thresholds for low (25–50 %), moderate (50–75 %) and high (>75 %) heterogeneity, respectively [10]. Meta-regression and subgroup analyses were performed to assess the potentially important covariates that might exert substantial impact on between-study heterogeneity [11]. We used the Egger regression asymmetry test to evaluate the publication bias [12]. Sensitivity analysis was conducted to describe how robust the pooled estimator was to removal of individual studies [13]. An individual study is suspected of excessive influence, if the point estimate of its omitted analysis lies outside the 95 % CI of the combined analysis. All statistical analyses were performed using Stata 12.0 (Stata Corp, College Station, Texas, USA). Two-tailed *P* ≤ 0.05 was accepted as statistically significant.

## Results

### Literature search

A total of 3558 citations were retrieved from the electronic databases. After initial screening of titles and abstracts using the aforementioned criteria, 45 articles were identified for full-text review (all the 45 articles were cited as a Additional file 1). Of these, 38 were further excluded, leaving seven eligible articles (Fig. 1). Hence, seven articles [14–20] involving 451 kidney stone cases and 482 controls were included in our final meta-analysis. Two studies were come from Iran, one from United States, one from Netherlands, one from Germany, one from Italy and one from Sweden. The characteristics of these included studies are presented in Table 1.

**Fig. 1:** The flow diagram of screened, excluded, and analyzed publications

**Table 1:** Characteristics of studies on the association between serum vitamin D levels and kidney stone risk

Study, year	Country	kidney stones assessed	Study type	Kidney stone			Controls		
				N (Male)	Age (Mean ± SD)	Serum vitamin D: Mean ± SD (ng/ml)	N (Male)	Age (Mean ± SD)	Serum vitamin D: Mean ± SD (ng/ml)
Berlin et al. [14]	Sweden	Symptomatic	Case-control	38 (34)	Na	26.2 ± 1.6	32 (16)	Na	17.6 ± 0.9
Fallahzadeh et al. [15]	Iran	Ultrasounds	Case-control	36 (24)	8.4 ± 4.7 months	33.85 ± 14.73	36 (22)	8.7 ± 4.7 months	18.26 ± 7.43
Giannini et al. [16]	Italy	Symptomatic	Case-control	25 (16)	41.2 ± 2.4	39.6 ± 2.6	15 (7)	49.0 ± 3.7	28.9 ± 1.8
Jarrar et al. [17]	Germany	Ultrasounds	Case-control	57 (35)	54.92 ± 23.32	53.65 ± 27.46	44 (22)	53.34 ± 18.51	48.3 ± 30.8
Leaf et al. [18]	United States	Ultrasounds	Randomized controlled trials	29 (22)	48 ± 12	35 ± 10	29 (22)	48 ± 12	17 ± 6
Netelenbos et al. [19]	Netherlands	Symptomatic	Case-control	160 (106)	43 ± 14	55 ± 23	217 (147)	39 ± 11	53 ± 22
Shakhssalim et al. [20]	Iran	Symptomatic	Case-control	106 (106)	43.4 ± 6.9	127 ± 40	109 (109)	38.4 ± 6.9	93 ± 35

*SD* standard deviation; *Na* not available

### Serum vitamin D level and kidney stone risk

Five of these included studies reported an increased risk of kidney stone for serum vitamin D levels in kidney stone patients compared with controls, while no significant association was reported in two studies. Our pooled results suggested that kidney stone patients had a significantly higher serum vitamin D level compared with non-kidney stone controls [summary SMD = 0.65, 95 % CI = 0.51, 0.79], with high between-study heterogeneity detected (I^2^ = 97.0 %, *P*_heterogeneity_ = 0.000) (Fig. 2).

**Fig. 2:** The forest plot of the association between serum vitamin D levels and kidney stone risk

#### Meta-regression and subgroup analysis

As seen in Fig. 2, evidence of high between-study heterogeneity (I^2^ = 97.0 %, *P*_heterogeneity_ = 0.000) was found in the pooled results. In order to explore the high between-study heterogeneity founded in the analysis, univariate meta-regression with the covariates of publication year, study design and geographic locations were performed. However, no significant findings were found in the above-mentioned analysis.

For the subgroup analyses by study design, the association was also significant in case–control studies [SMD = 0.57, 95 % CI = 0.43, 0.72; I^2^ = 97.2 %] of serum vitamin D levels in kidney stone patients compared with the controls. There is only one study was randomized controlled trials design, and no pooled results for other study design was combined. In subgroup analyses of geographic locations, when we restricted the analysis to Europe and Asia, the associations were significant both in European populations [SMD = 0.35, 95 % CI = 0.17, 0.53; I^2^ = 98.1 %] and in Asian populations [SMD = 1.00, 95 % CI = 0.76, 1.25; I^2^ = 51.4 %].

### Sensitivity analysis and publication bias

Sensitivity analysis showed that no individual study had excessive influence on the association of serum vitamin D levels with the risk of kidney stone. Egger’s regression asymmetry test (*P* = 0.596) showed no evidence of significant publication bias between serum vitamin D levels and kidney stone risk.

## Discussion

In this study, data were available with 451 kidney stone cases and 482 controls for the analysis. This work provided convincing evidence that serum vitamin D level in kidney stone patients was significantly higher than that in non-kidney stone controls. The associations were also significant both in Europe and in Asia populations.

In our study, significant between-study heterogeneity was found between serum vitamin D levels and kidney stone risk. Previous paper [21] had reported that heterogeneity is common in the meta-analyses. To explore the potential sources of between-study heterogeneity is therefore an essential component of meta-analysis. The high degree of heterogeneity might have arisen from publication year, study design and geographic locations. Therefore, we used meta-regression to explore the causes of heterogeneity by covariates. However, no covariate had significant impact on the high between-study heterogeneity among those mentioned above. Considering the pooled meta-analysis was fraught with the problem of heterogeneity, subgroup analyses by study design and geographic locations to explore the source of heterogeneity. However, between-study heterogeneity persisted in some of the subgroups, suggesting the presence of other unknown confounding factors. Other environment variables, as well as their possible interaction, may well be potential contributors to the heterogeneity observed.

As a meta-analysis of published studies, our findings showed some advantages. First, a highlight of this study was that we found a significant association between serum vitamin D levels and the risk of kidney stone. Second, the current study included more kidney stone cases and controls; this may derive a more precise estimation of the relationship between serum vitamin D and kidney stone risk. Third, no significant publication bias was detected in this meta-analysis.

There are some limitations in this meta-analysis should be concerned. First, six of the seven studies were case–control design and only one study was randomized controlled trials design. Although case–control studies may suffer from recall bias and selection bias, case–control studies are important methods in etiology research. More studies with other study design are wanted in the future studies. Second, as a meta-analysis of epidemiologic studies, we cannot rule out that individual studies may have failed to control for potential confounders, which may introduce bias in an unpredictable direction. Third, for the subgroups of geographic locations, the associations were significant both in Europe and in Asia between serum vitamin D levels and kidney stone risk. Only one study was conducted from United States. Thus, we did not combine the results for other populations. Due to this limitation, the results are applicable to Europe and Asia, but cannot be extended to other populations. More studies originating in other countries are required to investigate the association between serum vitamin D levels and kidney stone risk. Finally, between-study heterogeneity was high in the pooled analysis, but the heterogeneity was not successfully explained by the subgroup analysis and meta-regression. However, other environment variables, as well as their possible interaction may be potential contributors to this disease-effect unconformity.

## Conclusions

Findings from this meta-analysis suggest that serum vitamin D level in kidney stone patients was significantly higher than that in controls.

## Additional file

Additional file 1: The potentially relevant articles identified for full-text review. (DOCX 74 kb)
